The article "Comparison of Warming Needle Moxibustion and Drug Therapy for Treating Knee Osteoarthritis: A Systematic Review and Meta-analysis" was retracted in 2023. Reasons: signs of a paper mill; suspected computer-generated content; unreliable results or conclusions; lack of ethics approval or compliance.

# Comparison of Warming Needle Moxibustion and Drug Therapy for Treating Knee Osteoarthritis: A Systematic Review and Meta-analysis

**DOI:** 10.1155/2022/3056109

**Published:** 2022-07-27

**Authors:** Juan Li, Haizhou Yang, Tianyan Hu

**Affiliations:** ^1^The First Affiliated Hospital of Soochow University, Suzhou 215006, China; ^2^Suzhou TCM Hospital Affiliated to Nanjing University of Chinese Medicine, Suzhou 215000, China

## Abstract

**Objective:**

To compare the efficacy of warming needle moxibustion (WNM) with that of drug therapy for treating knee osteoarthritis (KOA), so as to provide evidence-based reference for the treatment of knee osteoarthritis.

**Methods:**

PubMed, Embase, Cochrane Library, VIP, WanFang, and CNKI were searched from inception to March 23, 2022. Literature selection was processed in strict accordance with inclusion and exclusion criteria. Cochrane Risk of Bias Assessment tool was applied for quality assessment of included studies. Data analysis and publication bias assessment were performed using Stata 15.0.

**Results:**

There were 30 RCTs included, with 1324 participants in the WNM group and 1293 in the control group. Meta-analysis showed that the WNM group yielded more excellent effect than the control group (*RR* = 1.22, 95% CI (1.17, 1.27), *p* = 0), improvement in WOMAC scores was greater in the WNM group than in the control group (WMD = −8.48, 95% CI (-13.13, -3.83), *p* = 0.002), activity of daily living (ADL) score was higher in the WNM group than in the control group (WMD = −7.66, 95% CI (-10.22, -5.09), *p* = 0.01), improvement in joint stiffness scores was greater in the WNM group than in the control group (WMD = -1.72, 95% CI (-2.50, -0.93), *p* = 0.005), and improvement in pain scores was greater in the WNM group than in the control group (SMD = −1.09, 95% CI (-1.38, -0.79), *p* = 0.001).

**Conclusions:**

WNM would be more effective in improving quality of life, decreasing WOMAC score, promoting knee function recovery, and alleviating the joint pain and stiffness, compared with orally taken drug therapies. Therefore, WNM could be given prior consideration for the treatment of KOA.

## 1. Introduction

Knee osteoarthritis (KOA) refers to a degenerative disease characterized by knee pain, movement disorder, and muscle dysfunction [1, 2] with high morbidity and incidence of joint deformity. It not only compromises patients' qualify of life but causes social-psychological problems such as anxiety, depression, sense of helplessness, and social dysfunction [3, 4] and brings heavy burden on their family and public health system [5]. Pathological features of KOA mainly include cartilage damage, osteophyte formation, and degenerations of subchondral bone and meniscus [6]. KOA is the primary type of meniscus, with high risk of disability, and the incidence in female is higher than that in male [7]. In traditional Chinese medicine, it seems almost inevitable that the morbidity will further increase, with the aging of population and the increasing numbers of obesity [8–10]. Conventional treatment for KOA is based on medications such as glucocorticoids and nonsteroidal anti-inflammatory drugs (NSAIDs), and surgery would be considered for severe cases, with a cost unaffordable for many patients [11]. Glucosamine hydrochloride is one of the primarily used agents for KOA while accompanied with many deficiencies such as relatively limited therapeutic effect, long treatment duration, susceptibility to drug dependence, and adverse reactions (diarrhea and drug eruption) [1, 12]. Therefore, exploration for safe and effective therapies from traditional Chinese medicine (TCM) is of great necessity. In recent years, great progress has been made in TCM for the treatment of KOA [13, 14].

The acupuncture and moxibustion methods for treating KOA include electric acupuncture, fire acupuncture, warming needle acupuncture, moxibustion, acupoint application, filiform acupuncture, and acuknife. Among them, warming needle acupuncture is one of the most commonly used methods. Warming needle moxibustion (WNM) is a therapeutic method that combines acupuncture and moxibustion, with efficacy of “channel-warming and cold-dispersing” and “blood-activating and stasis-eliminating” [15, 16]. Studies have demonstrated that WNM is one of the primary approaches for KOA treatment in China, and the potential mechanisms might be associated with the deceleration of knee cartilage degeneration [17–19], the regulation of inflammatory cytokines, and the reduction of algogenic substance release. A meta-analysis by Guo and Chen [20] proposed that more multicenter randomized controlled trials (RCTs) with large sample size and high quality are needed to further validate the efficacy of WNM for the treatment of KOA. Though increasing RCTs in this field have been conducted currently, there are many disputes on the efficacy of WNM and drug therapy [21–24]. We performed this systematic review and meta-analysis to compare the efficacy of WNM with drug therapy in expectation of providing evidence-based support for the application of WNM in clinical KOA treatment.

## 2. Materials and Methods

### 2.1. Inclusion and Exclusion Criteria

#### 2.1.1. Types of Study

The literatures reviewed and analyzed in this manuscript are based on randomized controlled trials (RCTs) results.

#### 2.1.2. Inclusion Criteria

Adults meet the diagnostic criteria of KOA. The experimental group took WNM as intervention, and the control group took oral medications of drug therapy. Outcome measures included overall therapeutic effect, knee function scores, the *Western Ontario and McMaster Universities* (WOMAC) *Osteoarthritis Index*, pain scores, joint stiffness scores, and activity of daily living scale (ADLs). Conference summaries, animal studies, reviews, repeated publication, and studies with data or full texts unavailable were excluded.

### 2.2. Literature Search

PubMed, Embase, Cochrane Library, VIP, WanFang, and China National Knowledge Infrastructure (CNKI) were searched, from inception to March 23, 2022, for RCTs regarding the comparison of WNM and drug therapy for the treatment of KOA. Search strategy was designed based on the combination of medical subject headings and free words, with search items containing “knee osteoarthritis,” “KOA,” “warming needle acupuncture,” “needle warming moxibustion,” “drug therapy,” etc.

### 2.3. Data Extraction

Literature selection and data extraction were conducted by two reviewers independently, and the results were cross-checked by each other. Any disagreements were settled through discussion with a third reviewer. Duplicates were removed followed by exclusion of irrelevant articles via browsing titles and abstracts, and the full texts of remaining articles were read to identify eligible studies.

Data extracted mainly included name of first author, publication date, study design, characteristics of participants, sample size, intervention and control, disease stage, and follow-up duration.

### 2.4. Quality Assessment

Quality assessment of included studies was performed by two reviewers independently using the Risk of Bias Assessment Tool provided in *Cochrane Handbook for Systematic Reviews of Interventions 5.1.0*, which contains seven domains: random sequence generation (selection bias), allocation concealment (selection bias), blinding of participants and personnel (performance bias), blinding of outcome assessment (detection bias), incomplete outcome data (follow-up bias), selective reporting (reporting bias), and other sources of bias. Each included study was assessed following the criteria mentioned above. Studies that fully met the criteria would be graded as “low risk,” indicating an overall low risk of bias, while those that partially met would be graded as “unclear risk,” indicating moderate risk of bias, and those fully unmet for the criteria as “high risk,” indicating high risk of bias and poor qualify of the studies.

### 2.5. Statistical Analysis

Meta-analysis was performed using Stata 16.0. Standard mean difference (SMD) and weighted mean difference (WMD) were applied as pooled statistics for continuous data, with 95% confidence intervals (95% CIs) provided. Risk ratio (RR) with 95% CI was used for dichotomous data. Heterogeneity test was conducted for each study. A *p* ≥ 0.1 with *I*^2^ < 50% indicated no significant heterogeneity existing between the studies, and fixed-effect model would be applied; otherwise (*p* < 0.1 with *I*^2^ ≥ 50%), significant heterogeneity would be considered, and subgroup analysis and sensitivity analysis would be conducted to identify the source of heterogeneity. Random-effect model would be used if the source of heterogeneity could not be identified. Publication bias was assessed using Begg's test, and a *p* > 0.05 indicated low risk of publication bias; otherwise, further sensitivity analysis would be performed to validate the robustness of the results.

## 3. Results

### 3.1. Literature Selection

There were 4932 articles identified, 2653 were retrieved after duplicate-checking, 2552 were excluded after title and abstract browsing, and 71 were excluded via full-text reading. A total of 30 RCTs were finally included. Detailed literature selection process is shown in Figure 1.

### 3.2. Characteristics of Included Studies

All the 30 included RCTs [21–50] were conducted in China. The experimental groups were WNM single intervention or WNM combined with TCM decoctions, and the control groups took oral drugs as intervention. There were a total of 1324 participants in the experimental group and 1293 in the control group, with the follow-up duration ranging from one to six months. Characteristics of included studies are shown in Table 1.

### 3.3. Quality Assessment of Included Studies

Quality assessment of included studies was performed by two reviewers independently using the Risk of Bias Assessment Tool provided in *Cochrane Handbook for Systematic Reviews of Interventions 5.1.0.* The overall quality was high, as shown in Table 2.

### 3.4. Results of Meta-analysis

#### 3.4.1. Therapeutic Effect

There were 24 studies [21–26, 28–32, 34–39, 41, 44, 46–50] that reported the therapeutic effect. Grouping was based on WNM or WNM+TCM decoctions versus orally taken drugs, with 1124 patients in the experimental group and 1029 in the control group. There was no significant heterogeneity between the studies (*I*^2^ = 41.7%, *p* = 0.018), and fixed-effect model was applied. Meta-analysis showed that compared with the control group, the WNM group yielded more excellent therapeutic effect, and the difference was statistically significant (*RR* = 1.22, 95% CI (1.17, 1.27), *p* = 0). WNM combined with TCM decoctions was also more effective, with significantly statistical difference (*RR* = 1.17, 95% CI (1.10, 1.25), *p* = 0.004), as shown in Figure 2.

#### 3.4.2. WOMAC Scores

There were 5 studies [26, 36, 37, 40, 50] that reported WOMAC scores, with 207 patients in the WNM group and 207 in the control group. There was significant heterogeneity considered (*I*^2^ = 83.8%, *p* = 0), and random-effect model was applied. Meta-analysis showed that the WNM group had more improved WOMAC scores than the control group, and the difference was statistically significant (WMD = −8.48, 95% CI (-13.13, -3.83), *p* = 0.002). Subgroup analysis showed that there was no difference in the improvement of WOMAC scores between the WNM group and control group (WMD = −8.88, 95% CI (-17.8, 0.03) *p* = 0.051), while WNM combined with TCM decoctions resulted in more improved WOMAC scores, compared with orally taken drugs (WMD = −7.70, 95% CI (-10.36, -5.05), *p* = 0.001, as shown in Figure 3.

#### 3.4.3. Joint Stiffness Scores

There were 5 studies [26, 28, 34, 37, 43] that reported joint stiffness scores, with 269 in the WNM group and 269 in the control group. There was significant heterogeneity considered (*I*^2^ = 61%, *p* = 0.036), and random-effect model was applied. Meta-analysis showed that the WNM group had more improved joint stiffness scores than the control group, and the difference was statistically significant (WMD = −1.72, 95% CI (-2.50, -0.93), *p* = 0.005), as shown in Figure 4.

#### 3.4.4. ADL Scores

There were 5 [26, 28, 34, 37, 43] studies that reported ADL scores, with 307 in the WNM group and 298 in the control group. There was significant heterogeneity considered (*I*^2^ = 56.2%, *p* = 0.058), and random-effect model was applied. Meta-analysis showed that patients in the WNM group had higher ADL scores than those in the control group, and the difference was statistically significant (WMD = -7.66, 95% CI (-10.22, -5.09), *p* = 0.01), as shown in Figure 5.

#### 3.4.5. Pain Scores

There were 14 studies [25–28, 31, 32, 35–37, 42, 43, 48–50] that reported changes in pain scores before and after treatment, with 841 in the WNM group and 823 in the control group. There was significant heterogeneity considered (*I*^2^ = 82.5%, *p* = 0), and random-effect model was applied. Meta-analysis showed that patients in the WNM group had more improved pain scores than those in the control group, and the difference was statistically significant (SMD = −1.09, 95% CI (-1.38, -0.79), *p* = 0.001). In subgroup of WNM combined with TCM decoctions, WNM was more effective in improving pain scores than orally taken drugs (SMD = −1.21, 95% CI (-1.79, -0.46), *p* = 0.0001). In subgroup of WNM, patients in the WNM group had more improved pains scores than those in the control group (SMD = −1.04, 95% CI (-1.39, -0.69), *p* = 0.003), as shown in Figure 6.

#### 3.4.6. Knee Function Scores

There were 5 studies that reported changes in knee function scores, with 345 in the WNM group and 345 in the control group. There was significant heterogeneity considered (*I*^2^ = 62.2%, *p* = 0.032), and random-effect model was applied. Meta-analysis showed that patients in the WNM group had less improved knee function scores than those in the control group, and the difference was statistically significant (SMD = 1.78, 95% CI (1.45, 2.12), *p* = 0), as shown in Figure 7.

### 3.5. Sensitivity Analysis

Sensitivity analysis was performed for the therapeutic effect and pain scores via removing the studies one by one. The results showed that the circles representing each study were within the two edges, indicating that results of meta-analysis were robust and reliable (see Figures 8 and 9).

### 3.6. Publication Bias

Begg's test was applied for the therapeutic effect and pain scores, to assess the publication bias. The *p* value of the therapeutic effect was 1.14, and that of pain scores was 0.155. Both the *p* values were greater than 0.05, suggesting a minimal possibility of publication bias (see Figures 10 and 11).

## 4. Discussion

The load of human body normally transmits along the alignment of lower limbs, from center of femur head to that of ankle joint, through center of knee joint or slightly medial of that. Abnormal alignment induced by multiple factors inside or outside knee joint could change the biomechanics of lower limb, leading to an uneven distribution of stress in the joint and subsequently articular cartilage damage, which underlies the primary biomechanical pathogenesis of KOA [51]. Wu et al. [52] acupunctured Neixiyan point (EX-LE4) and Waixiyan point (ST35) of KOA patients for 4 weeks and found that the peak torque, relative peak torque, fatigue index, and the corresponding angle of peak torque of these patients were significantly improved, which revealed that acupuncture could improve the strength of muscles around knee joint and rebalance their biomechanics and could increase the suppleness and stability of knee joint, so that symptoms attenuate. Decline and imbalance of muscle strength commonly exists in the quadriceps femoris and hamstrings of KOA patients, which is closely related to their joint pain and limited function. Muscles are important for body vibration absorption, and proper strength and balance of flexors and extensors around knee joint (mainly refer to quadriceps femoris and hamstrings) are of essence for maintaining joint stability [53]. The joint pain and limited joint movement accompanied with decreased muscle strength in KOA patients compromise the joint stability, increase the load, and shift its movement mode, which causes imbalanced internal stress and aggravates cartilage degeneration [54, 55]. KOA belongs to the category of “Bi” syndrome in TCM. *Huangdi's Internal Classic Plain Question* proposed that the mix of wind, cold, and dampness induces the Bi syndrome. *Zhangshi Yitong* stated that knee is the house of muscles, and there is no knee pain without the involvement of liver and kidney deficiency in that wind, cold, and dampness set in under the deficiency [13]. Ancient TCM practitioners had a consistent sense of the disease. The locations of the disease are in the liver, kidney, muscle, and bone, the nature of that is deficiency in origin and excess in symptoms, and the pathogenesis includes liver and kidney deficiency, muscle and bone malnutrition, rise of cold due to Yang deficiency, and phlegm-stasis blocking collateral [56, 57]. Acupuncture has the effect of regulating qi and replenishing blood, and to clear and activate the channels and collaterals, and that of moxibustion to stimulate the circulation of the blood and cause the muscles and joints to relax, and relieve depression and pain. WNM is a therapeutic method that combines acupuncture and moxibustion, by which the heat of moxibustion is transmitted along the needle body and from the handle to acupoints, so as to produce warm stimulation to human body. Its acting on acupoints grant it remarkable effect of channel-warming, cold-dispersing and relieve the pain and tension. Conventional drug therapy has effects of anti-inflammation and pain-relief and has been widely applied to alleviate the pain symptoms in KOA patients, while these agents have adverse reactions like gastrointestinal reaction. It is reported that several new NSAIDs, such as COX-2 inhibitors, have relatively mild gastrointestinal reaction but have risk for cardiovascular events [58, 59].

We found that the WNM group yielded more excellent effect than the control group (*RR* = 1.22, 95% CI (1.17, 1.27), *p* = 0), improvement in WOMAC scores was greater in the WNM group than in the control group (WMD = −8.48, 95% CI (-13.13, -3.83), *p* = 0.002), ADL score was higher in the WNM group than in the control group (WMD = −7.66, 95% CI (-10.22, -5.09), *p* = 0.01), improvement in joint stiffness scores was greater in the WNM group than in the control group (WMD = −1.72, 95% CI (-2.50, -0.93), *p* = 0.005), and improvement in pain scores was greater in the WNM group than in the control group (SMD = −1.09, 95% CI (-1.38, -0.79), *p* = 0.001). This is consistent with the results of the study by Hong et al. [60], which used WNM to treat 30 KOA patients with TCM syndrome of cold-congealing due to Yang deficiency. They chose Neixiyan point (penetrating onto outer top) and Waixiyan point (penetrating onto inner top) as main acupoints and implemented two “Zhuang” of moxibustion for each regimen. The WNM group resulted in greater therapeutic effect than the control group. Yu [61] applied WNM to treat 32 KOA cases. Yu chose Neixiyan (EX-LE4), Waixiyan (ST 35), Liangqiu (ST 34), Xuehai (SP 10), Yinlingquan (SP 9), Yanglingquan (GB 34), and Zusanli (ST 36), as treatment points in the WNM group, and used acupuncture alone as control, with the same acupoints as the WNM group. Both the two groups were treated once a day for 2 treatment courses (10 days as a treatment course). The WNM group resulted in an effective rate of 96.9% greater than the control group. These studies demonstrated that WNM could improve local blood circulation, promote joint repair, relieve the symptoms, and alleviate joint pain in the treatment of KOA. Acupuncture directly acts on the lesion area and the nearby acupoints, which could not only stimulate nerve terminals and their receptors to send impulses to the high-level center, so as to promote systemic or local response, but promote the conduction of acupuncture sensations through affecting the meridian system so that produce systemic and local effects. The combination with moxibustion presents a positively regulating effect on the secretion of matrix metalloproteinases and their inhibitors in arthritis synovial cells.

This study has the following limitations: first, the included studies were all Chinese studies and published in Chinese, which may affect the conclusion of this study. Second, most studies do not describe blindness, which may lead to methodological bias. Finally, the acupoints used in each study are different and the control drugs are also different, which may lead to a greater risk of deviation in our paper.

## 5. Conclusion

In China, WNM is more effective in improving quality of life, reducing WOMAC score, promoting functional recovery of the knee joint, and relieving joint pain and stiffness compared with drug therapy. Therefore, WNM can be prioritized for the treatment of KOA. Given the limitations of the included studies, more large-sample, high-quality multicenter RCTs are needed.

## Figures and Tables

**Figure 1:** Flow diagram of literature selection.

**Figure 2:** Forest plot of the therapeutic effect.

**Figure 3:** Forest plot of WOMAC scores.

**Figure 4:** Forest plot of joint stiffness scores.

**Figure 5:** Forest plot of ADL scores.

**Figure 6:** Forest plot of improvement in pain scores.

**Figure 7:** Forest plot of improvement in knee function scores.

**Figure 8:** Sensitivity analysis for the therapeutic effect.

**Figure 9:** Sensitivity analysis for pain scores.

**Figure 10:** Publication bias plot of the therapeutic effect.

**Figure 11:** Publication bias plot of pain scores.

**Table 1:** Characteristics of included studies.

First author	Year	Type of research	Intervention		Number of cases		Gender (male/female)		Age (years old)		Disease grading/staging	Follow-up time
			Experimental group	Control group	Experimental group	Control group	Experimental group	Control group	Experimental group	Control group	/	
Shanghua Xia	2018	RCT	Traditional Chinese medicine: take by mouth and wash externally (different medication for patients with different symptoms), plus acupuncture	Drug therapy treatments and approaches (not specified)	40	40	/	/	71.66 ± 2.15	70.95 ± 2.58	/	/
Wei Lijuan	2019	RCT	Traditional Chinese medicine: take by mouth and wash externally (different medication for patients with different symptoms), plus acupuncture	Drug therapy treatments and approaches (not specified)	40	40	/	/	/	/	/	1 month
He Caiyuan	2017	RCT	Warming needle moxibustion	300 mg Fenbid capsule (ibuprofen sustained release capsule)	42	42	22/20	23/19	66.2 ± 6.3	67.5 ± 6.1	Experimental group (28 cases reporting single knee pain of onset and 14 cases reporting bilateral knee pain of onset) Control group (26 cases reporting single knee pain of onset and 16 cases reporting bilateral knee pain of onset)	/
Tang Yu	2020	RCT	Warming needle moxibustion	1 tablet/d meloxicam oral	49	49	28/21	30/19	60.8 ± 9.2	61.5 ± 8.5	Experimental group: average pathogenesis 2.7 ± 1.0 Control group: average pathogenesis 2.6 ± 1.1	1 month
Liu Si	2021	RCT	Warming needle moxibustion	2 capsules/d Fenbid capsule	39	39	21/18	23/16	63.41 ± 6.12	63.69 ± 6.17	Experimental group: average pathogenesis 4.65 ± 1.71 Control group: average pathogenesis 4.93 ± 1.78	28 d
Han Naiyi	2021	RCT	Warming needle moxibustion	1 capsule/d ibuprofen sustained release capsule	37	37	/	/	58.89 ± 5.67	58.91 ± 5.77	Experimental group: average pathogenesis 5.41 ± 2.19 Control group: average pathogenesis 5.37 ± 2.23	
Wang Xiongwei	2021	RCT	Warming needle moxibustion	Injecting sodium hyaluronate into articular cavity	36	36	20/16	22/14	59.92 ± 6.03	59.98 ± 6.14	Experimental group: average pathogenesis 3.58 ± 1.29 Control group: average pathogenesis 3.49 ± 1.17	1 month
He Nanxia	2020	RCT	Warming needle moxibustion	Ibuprofen sustained release capsule	21	21	12/9	11/10	57.62 ± 4.51	57.48 ± 4.63		
Zheng Wenjie	2012	Quasi-RCT	Warming needle moxibustion plus fumigation-washing therapy	0.4 g/d meloxicam capsule	48	30	12/36	11/19	50.62 ± 8.96	51 ± 9.26	Experimental group: average pathogenesis 3.69 ± 3.12 Control group: average pathogenesis 3.76 ± 2.86	1 month
Huang Yanxi	2013	RCT	Warming needle moxibustion plus flash cupping therapy	Celebrex oral plus topical TDP lamp therapy	60	60	28/32	26/31	55.13 ± 11.2	55.15 ± 10.3	Experimental group (38 cases reporting single knee pain of onset and 22 cases reporting bilateral knee pain of onset) Control group (37 cases reporting single knee pain of onset and 20 cases reporting bilateral knee pain of onset)	20 d
Lei Bo	2016	RCT	Warming needle moxibustion plus decoction	Glucosamine hydrochloride capsules	30	30	15/15	16/14	57.6 ± 2.6	58.5 ± 1.8	Experimental group (16 cases reporting single knee pain of onset and 14 cases reporting bilateral knee pain of onset) Control group (16 cases reporting single knee pain of onset and 14 cases reporting bilateral knee pain of onset)	1 month
Qiu Sheng	2013	RCT	Warming needle moxibustion	1 capsule/d ibuprofen sustained release capsule	36	38	15/21	17/21	55.5 ± 5.6	56.6 ± 6.2	Experimental group: average pathogenesis 12.3 ± 2.3 yrs Control group: average pathogenesis 12.2 ± 2.5	1 month
Zhou Miao	2015	RCT	Warming needle moxibustion	75 mg/d Voltaren	38	29	22/16	18/11	50.59 ± 4.73	49.73 ± 4.29	Experimental group: average pathogenesis 5.12 ± 0.76 Control group: average pathogenesis 5.03 ± 0.77	9 weeks
Xu Hongbing	2020	RCT	Warming needle moxibustion	0.3 mg/d ibuprofen sustained release capsule	55	55	28/27	29/26	53.8 ± 4.77	53.91 ± 4.63	Experimental group: average pathogenesis 1.88 ± 0.53 Control group: average pathogenesis 1.76 ± 0.51	1 month
Shu Yan	2021	RCT	Warming needle moxibustion	1 tablet/d diclofenac sodium sustained release tablets	30	30	20/10	19/11	62.5 ± 5.1	64.5 ± 5.3	Experimental group: average pathogenesis 6.2 ± 0.5 Control group: average pathogenesis 7.3 ± 0.7	28 d
Ren Zhenjia	2018	RCT	Warming needle moxibustion	6 tablets/d take glucosamine hydrochloride tablets by mouth	54	54	23/31	25/29	67.1 ± 4.6	68.7 ± 5.2	Experimental group: average pathogenesis 4.9 ± 1.5 Control group: average pathogenesis 4.6 ± 1.7	6 months
Yang Wenwu	2020	RCT	Warming needle moxibustion	Ibuprofen sustained release capsule	34	34	21/47		58.23 ± 7.12		4.58 ± 1.29	
Gao Xiaobo	2020	Quasi-RCT	Warming needle moxibustion	Sodium hyaluronate	44	44	24/20	23/21	55.45 ± 10.25	55.36 ± 10.32	Experimental group: average pathogenesis 10.34 ± 8.11 Control group: average pathogenesis 10.03 ± 8.56	6 months
Ming Hui	2009	RCT	Warming needle moxibustion	Ibuprofen sustained release capsule	30	30	8/22	9/21	59.37 ± 12.2	52.03 ± 16.10	Experimental group: average pathogenesis 50.23 ± 47.5 months Control group: average pathogenesis 62.2 ± 45.67	10 weeks
Wu Yongli	2006	RCT	Warming needle moxibustion	75 mg/d Voltaren	60	54	23/37	15/39	38-82	40-78		20 d
He Zhengyu	2016	RCT	Warming needle moxibustion	2 capsules/d ibuprofen sustained release capsule	62	62	32/30	35/27	63.3 ± 4.1	61.8 ± 4.3		30 d
Cai Xia	2020	RCT	Warming needle moxibustion	Ibuprofen sustained release capsule	75	75	41/34	43/32	57.3 ± 4.5	56.7 ± 4.7	Experimental group: average pathogenesis 5.5 ± 1.2 yrs Control group: average pathogenesis 5.4 ± 1.3	2 weeks
Yao Xiaobing	2018	RCT	Warming needle moxibustion	0.6 g/d ibuprofen sustained release capsule	40	40	12/18	11/19	61.2 ± 4.5	62.4 ± 4.8		8 weeks
Tai Xinhua	2016	RCT	Warming needle moxibustion	Glucosamine sulfate tablets	30	30	13/17	15/15	68.4 ± 2.9	67.9 ± 2.7		2 months
He Zhiqian	2019	RCT	Warming needle moxibustion	0.6 g/d ibuprofen tablet	29	29	15/14	16/13	51.02 ± 5.98	51.21 ± 5.77		10 d
Xu Hongbing	2014	RCT	Warming needle moxibustion	Diclofenac sodium sustained release tablets	30	30	32/28		68.3 ± 5.9		Average pathogenesis 11.2 ± 3.5 yrs	2 weeks
Lei Anjun	2020	RCT	Warming needle moxibustion	Diclofenac sodium sustained release tablets	53	53	18/35	20/33	58.09 ± 10.22	58.13 ± 10.18	Experimental group: average pathogenesis 31.87 ± 2.09 months Control group: average pathogenesis 31.69 ± 2.11	1 month
Wang Tianzi	2021	RCT	Decoction of Angelica sinensis for warming cold limbs plus warming needle moxibustion	0.2 g/d take meloxicam capsule by mouth	108	108	57/51	58/50	59.2 ± 3.27	59.12 ± 3.25	Experimental group: average pathogenesis 2.4 ± 0.52 yrs Control group: average pathogenesis 2.36 ± 0.57	6 weeks
Pan Qihua	2022	RCT	Decoction of angelica sinensis for warming cold limbs plus warming needle moxibustion	0.2 g/d take meloxicam capsule by mouth	30	30	13/17	11/19	62.11 ± 10.03	63.79 ± 9.92	Experimental group: average pathogenesis 4.91 ± 1.69 yrs Control group: average pathogenesis 5.01 ± 1.72	6 weeks
Zhi Jianlong	2019	RCT	Decoction of angelica sinensis for warming cold limbs plus warming needle moxibustion	0.2 g/d meloxicam capsule	44	44	17/27	19/25	63.19 ± 7.73	62.52 ± 8.13	Experimental group: average pathogenesis 5.16 ± 2.34 yrs Control group: average pathogenesis 4.94 ± 2.06	6 weeks

**Table 2:** Quality assessment of included studies.

Study	Random sequence generation	Allocation concealment	Blinding of participants and personnel	Blinding of outcome assessment	Incomplete outcome data	Selective reporting	Other bias
Xia Shanghua 2018	High	Unclear	Unclear	Unclear	Low	Low	Unclear
Wei Lijuan 2019	Low	Unclear	Unclear	Unclear	Low	Low	High
He Caiyuan 2017	High	Unclear	Unclear	Unclear	Low	Low	Unclear
Tang Yu 2020	Low	Unclear	Unclear	Unclear	Low	Low	Unclear
Liu Si 2021	Low	Unclear	Unclear	Unclear	Low	Low	Unclear
Han Naiyi 2021	Low	Unclear	Unclear	Unclear	Low	Low	Unclear
Wang Xiongwei 2021	Low	Unclear	Unclear	Unclear	Low	Low	Unclear
He Nanxia 2020	Low	Unclear	Unclear	Unclear	Low	Low	Unclear
Zheng Wenjie 2012	High	Unclear	Low risk	Unclear	Low	Low	Unclear
Huang Yanxi 2013	Low	Unclear	Unclear	Unclear	Low	Low	Unclear
Lei Bo 2016	Low	Unclear	Unclear	Unclear	Low	Low	Unclear
Qiu Sheng 2013	Low	Unclear	Unclear	Unclear	Low	Low	High
Zhou Miao 2015	Unclear	Unclear	Unclear	Unclear	Low	Low	Unclear
Xu Hongbing 2020	Unclear	Unclear	Unclear	Unclear	Low	Low	Unclear
Shu Yan 2021	Unclear	Unclear	Unclear	Unclear	Low	Low	Unclear
Ren Zhenjia 2018	Low	Unclear	Unclear	Unclear	Low	Low	Unclear
Yang Wenwu 2020	Unclear	Unclear	Unclear	Unclear	Low	Low	Unclear
Gao Xiaobo 2020	High	Unclear	Unclear	Unclear	Low	Low	Unclear
Ming Hui 2009	Low	Unclear	Unclear	Unclear	Low	Low	Unclear
Wu Yongli 2006	Unclear	Unclear	Unclear	Unclear	Low	Low	Unclear
He Zhengyu 2016	Unclear	Unclear	Unclear	Unclear	Low	Low	Unclear
Cai Xia 2020	Unclear	Unclear	Unclear	Unclear	Low	Low	Unclear
Yao Xiaobing 2018	Low	Unclear	Unclear	Unclear	Low	Low	Unclear
Tai Xinhua 2016	Unclear	Unclear	Unclear	Unclear	Low	Low	Unclear
He Zhiqian 2019	Low	Unclear	Unclear	Unclear	Low	Low	High
Xu Hongbing 2014	Unclear	Unclear	Unclear	Unclear	Low	Low	Unclear
Lei Anjun 2020	Unclear	Unclear	Unclear	Unclear	Low	Low	Unclear
Wang Tianzi 2021	Low	Unclear	Unclear	Unclear	Low	Low	Unclear
Pan Qihua 2022	Low	Unclear	Unclear	Unclear	Low	Low	Unclear
Zhi Jianlong 2019	Unclear	Unclear	Unclear	Unclear	Low	Low	Unclear

## Data Availability

The data used to support the findings of this study are included within the article.
